# Impact of delivery mode on the colostrum microbiota composition

**DOI:** 10.1186/s12866-017-1109-0

**Published:** 2017-09-25

**Authors:** Marco Toscano, Roberta De Grandi, Diego Giampietro Peroni, Enzo Grossi, Valentina Facchin, Pasquale Comberiati, Lorenzo Drago

**Affiliations:** 1 Laboratory of Clinical Microbiology, Department of Biomedical Sciences for Health, University of Milan, Via Mangiagalli 31, Milan, 20133 Italy; 2 Department of Clinical and Experimental Medicine, Section of Pediatric and International Inflammation (in-FLAME) Network of the World Universities Network, University of Pisa, Pisa, Italy; 3 Villa Santa Maria Institute, Via IV Novembre Tavernerio, 22038 Como, Italy; 4 Department of Surgical Sciences, Dentistry, Gynecology and Pediatrics, Section of Pediatrics, University of Verona, Verona, Italy; 5 Laboratory of Clinical-Chemistry and Microbiology, IRCCS Galeazzi Institute, University of Milan, Via R. Galeazzi 4, 20164 Milan, Italy

**Keywords:** Microbiota, Colostrum, Breast milk, Bacteria, Network, Auto contractive map

## Abstract

**Background:**

Breast milk is a rich nutrient with a temporally dynamic nature. In particular, numerous alterations in the nutritional, immunological and microbiological content occur during the transition from colostrum to mature milk. The objective of our study was to evaluate the potential impact of delivery mode on the microbiota of colostrum, at both the quantitative and qualitative levels (bacterial abundance and microbiota network).

**Methods:**

Twenty-nine Italian mothers (15 vaginal deliveries vs 14 Cesarean sections) were enrolled in the study. The microbiota of colostrum samples was analyzed by next generation sequencing (Ion Torrent Personal Genome Machine). The colostrum microbiota network associated with Cesarean section and vaginal delivery was evaluated by means of the Auto Contractive Map (AutoCM), a mathematical methodology based on Artificial Neural Network (ANN) architecture.

**Results:**

Numerous differences between Cesarean section and vaginal delivery colostrum were observed. Vaginal delivery colostrum had a significant lower abundance of *Pseudomonas* spp., *Staphylococcus* spp. and *Prevotella* spp. when compared to Cesarean section colostrum samples. Furthermore, the mode of delivery had a strong influence on the microbiota network, as Cesarean section colostrum showed a higher number of bacterial *hubs* if compared to vaginal delivery, sharing only 5 *hubs*. Interestingly, the colostrum of mothers who had a Cesarean section was richer in environmental bacteria than mothers who underwent vaginal delivery. Finally, both Cesarean section and vaginal delivery colostrum contained a greater number of anaerobic bacteria genera.

**Conclusions:**

The mode of delivery had a large impact on the microbiota composition of colostrum. Further studies are needed to better define the meaning of the differences we observed between Cesarean section and vaginal delivery colostrum microbiota.

## Background

Human colostrum is a rich nourishing substance that is essential for the initial development of newborns [1]. Colostrum is produced by the mammary glands starting immediately after delivery until the fifth/sixth day of the newborn’s life; it is rich in cytokines, antimicrobial peptides, mineral salts, antibodies, hormones and bioactive factors with a strong immunomodulatory activity [1–4]. Consequently, the ingestion of colostrum represents not only the fundamental source of nutritive elements but also a way for infants to adapt to the extra-uterine environment [5]. Moreover, colostrum reduces the risk of gastrointestinal diseases, such as necrotizing enterocolitis, mitigates inflammatory responses and influences the gut microbiota composition of newborns [2, 6–8]. Colostrum and also mature milk represent an important source of bacteria, more than 200 different species, which have a strong impact on the newborn’s health for up to several months after birth [9]. Colostrum contains numerous microorganisms including *Staphylococcus*, *Streptococcus* and *Bacteroides* genera, that together with probiotic bacteria such as *Alloiococcus* spp., can reduce the incidence and severity of several gastrointestinal infections by both competitive exclusion mechanisms and production of antimicrobial compounds [1, 10]. Interestingly, the transition from colostrum to mature milk influences the bacterial composition, as changes in the abundance of several microorganisms, together with a significant modification of bacterial interactions (microbiota network) have been detected [9]. These findings highlight the extreme dynamic nature of human breast milk as a result of external and internal influences. Although the specific mechanisms involved in the origin of colostrum and mature milk microbiota are still under investigation, two main hypotheses exist: i) the existence of an entero-mammary pathway, which could lead intestinal bacteria directly to the mammary ducts by means of dendritic cells and CD18^+^ cells; ii) a retrograde flow during nursing whereby the oral bacteria of infants could influence the colostrum microbiota [9, 11].

Interestingly, a recent study also highlighted the potential role that the mode of delivery can have in modulating the bacterial composition of human mature milk, as the concentration of various bacterial genera was higher in the breast milk of mothers who underwent vaginal delivery as opposed to mothers who underwent Cesarean section (C-section) [12]. Recently, the effects of C-section versus vaginal delivery on the composition of infant microbiota and on infant health have been the object of numerous studies and yet, the specific effects they have on human life have not been fully clarified [13–15].

The aim of the present study was to assess the effect of delivery mode on the microbiota composition of colostrum samples. Specifically, we evaluated both bacterial abundance and interactions (microbiota network) within colostrum samples associated with either C-section or vaginal delivery by a next generation sequencing (NGS) approach applied to Auto-Contractive Map (AutoCM).

## Results

### Bacterial diversity in the colostrum microbiota in relation to the mode of delivery

To evaluate any differences in the bacterial diversity between the colostrum belonging to mothers who underwent natural delivery and mothers who delivered by C-section, we calculated the Shannon, Simpson and Chao’s indices (Fig. 1). Although no significant differences in biodiversity was observed, colostrum associated with natural delivery had a higher biodiversity compared to C-section colostrum. Both Shannon and Chao’s indices were slightly higher in natural delivery colostrum (Fig. 1).

**Fig. 1:** Shannon, Simpson and Chao’s indices of C-section and vaginal delivery colostrum. Non-parametric Kruskal-Wallis test was used to find significant differences in α diversity. No significant differences in biodiversity were observed, even if colostrum associated with natural delivery had a higher biodiversity compared to C-section colostrum

### Bacterial differences in colostrum microbiota in relation to the mode of delivery

Several significant differences were observed comparing the microbiota composition of C-section colostrum with that of vaginal delivery (Fig. 2). In particular, the latter was significantly richer in microorganisms belonging to *Streptococcus* and *Haemophilus* genera (more abundant by approximatively 49% and 94%, respectively), with a significant lower abundance of *Finegoldia* spp. (approximately 94%), *Halomonas* spp. (approximately 70%), *Prevotella* spp. (approximately 74%), *Pseudomonas* spp. (69%) and *Staphylococcus* spp. (approximately 29%) (Fig. 2).

**Fig. 2:** Significant differences in bacterial abundance between C-section and vaginal delivery colostrum (*p* value <0.05). Mann-Whitney test was used to find significant differences in microbial taxa between different samples. *P*-values below 0.05 were considered statistically significant

### Abundance of anaerobic and aerobic bacteria in colostrum samples

On one hand, both C-section and vaginal delivery colostrum contained a higher number of anaerobic than aerobic bacterial genera (approximately 65% anaerobic genera) (Fig. 3a). However, a greater absolute number of aerobic microorganisms were observed in all colostrum samples for each single genus (Fig. 3b). Interestingly, C-section colostrum showed a greater number of environmental microorganisms compared to vaginal delivery colostrum (Fig. 4a). Finally, both C-section and vaginal delivery colostrum showed a high abundance of intestinal bacterial genera (Fig. 4b).

**Fig. 3:** **a** Percentage distribution of aerobic and anaerobic bacterial genera in both C-section and vaginal delivery colostrum; **b** Relative abundance (total reads) of aerobic and anaerobic bacteria contained in colostrum samples

**Fig. 4:** **a** Percentage of environmental bacterial genera contained in colostrum samples; **b** Percentage of intestinal bacterial genera in both C-section and vaginal delivery colostrum samples. To identify environmental bacteria in the colostrum microbiota we used different online free tools (see Methods) that allowed the characterization of the majority of microorganisms contained in colostrum

### Colostrum bacterial networks (AutoCM)

The main interactions between bacteria detected in C-section and vaginal delivery colostrum were identified using AutoCM, by linking all the variables considered. The AutoCM matrix was then filtered by a minimum spanning tree algorithm (MST) which maps only the strongest correlations between the system hubs connected to a node. Only a single path is available between two hubs, without formation of loops (1). Microorganisms showing at least three connections with other microbes in the network were considered as the main bacterial *hubs*.

We found numerous differences between the colostrum networks of C-section and vaginal delivery samples. In detail, the main bacterial *hubs* of C-section colostrum were *Achromobacter*, *Acinetobacter*, *Aerococcus*, *Akkermansia*, *Amaricoccus*, *Anaerococcus*, *Aquabacterium*, *Butyriricimonas*, *Delftia*, *Dermabacter*, *Enterobacter*, *Haemophilus*, *Pectobacterium*, *Peptostreptococcus*, *Rhizobium*, *Rhodanobacter*, *Roseburia*, *Ruminococcus*, *Serratia*, *Staphylococcus* and *Sutterella* (Fig. 5). The central nodes of this network were represented by *Ruminococcus* and *Peptostreptococcus*.

**Fig. 5:** Microbiota network of C-section colostrum. Red circles represent all bacterial hubs identified in the colostrum microbiota. Microorganisms showing at least three connections with other microbes in the network were considered as the main bacterial *hubs*

The vaginal delivery colostrum, instead, showed a different microbiota network in which the main *hubs* were represented by *Achromobacter, Aeromonas, Bacillus*, *Blautia*, *Clostridium*, *Coprococcus*, *Eubacterium*, *Faecalibacterium*, *Granulicatella*, *Kocuria*, *Micrococcus*, *Oscillibacter*, *Rhodanobacter*, *Raoultella*, *Ruminococcus*, *Serratia* and *Staphylococcus* (Fig. 6). The central nodes of this network were *Rhodanobacter* and *Achromobacter*; the latter also represents the bacterial *hub* with more interactions with other microorganisms (16 connections).

**Fig. 6:** Microbiota network of vaginal delivery colostrum. Red circles represent all bacterial hubs identified in the microbiota colostrum. Microorganisms showing at least three connections with other microbes in the network were considered as the main bacterial *hubs*

Only the *hubs Achromobacter*, *Rhodanobacter*, *Ruminococcus*, *Serratia* and *Staphylococcus* were shared between the two colostrum microbiota networks.

## Discussion

Colostrum is known to be a dynamic biological sample which changes its nutritional and microbiological composition over time [1]. Diet is one of the main factors which can influence the composition of colostrum microbiota and for this reason all mothers enrolled in the present study had the same dietary intake, namely a large amount of animal proteins, fat and sugar in their diet.

In the present study, the colostrum microbiota composition was strongly influenced by the mode of delivery, as significant differences in terms of biodiversity, bacterial abundance and microbial interactions were observed comparing C-section colostrum microbiota with that of vaginal delivery. In particular, colostrum belonging to mothers who underwent vaginal delivery showed a slightly greater bacterial richness if compared to C-section colostrum. Generally, bacterial diversity promotes the maintenance and improvement of a balanced environment; an ecosystem with greater biodiversity, which is richer in bacterial species, is more resilient and adaptable to stress than one with a low range of microorganisms [16]. Moreover, vaginal delivery colostrum was observed to be significantly richer in microorganisms belonging to *Streptococcus* and *Haemophilus* genera, both of which include commensal and pathogenic microorganisms. *Haemophilus* is generally considered an opportunistic pathogen with a negative role on the host’s health [17]; although we observed that *Haemophilus* was more abundant in vaginal delivery colostrum, it was of crucial importance only in C-section colostrum where it acted as one of the main bacterial *hubs* detected in the microbiota network. Furthermore, in this microbiota network *Haemophilus* was strictly connected to *Peptostreptococcus* spp., *Achromobacter* spp. and *Kluyvera* spp. whose involvement in human skin and tissue infections have already been observed [18–20]. The aforementioned interaction implies a potential biological correlation between these four bacterial genera that may have a deeper impact on the host’s health than the significant greater abundance of *Haemophilus* spp. detected in vaginal delivery colostrum. This result is of great significance as it supports the idea that the pathogenicity of a microorganism is not always associated to its abundance in the environment, but rather it involves several factors including interactions with others microbes.

Considering all bacterial *hubs* detected in both C-section and vaginal delivery colostrum, the former showed a higher abundance of microorganisms of environmental origin if compared to the latter. Probably, mothers undergoing C-section are more exposed to environmental bacteria; this could play a pivotal role in modulating the microbiota of colostrum. It has already been demonstrated that C-section significantly influences the composition of intestinal microbiota in the early stages of human life, as newborns are primarily subjected to environmental bacteria that can lead to a decrease in bacterial diversity and richness [21]. Therefore, it is reasonable to hypothesise that also the mothers’ microbiota, including that of the colostrum, is strongly influenced by environmental microorganisms acquired by the infant, during childbirth. More interestingly, both kinds of colostrum samples analyzed in the present study contained a high percentage of intestinal microorganisms, this strengthens the entero-mammary hypothesis, which states that the microbiota of the colostrum is strongly influenced by the host’s own intestinal bacteria [22–25]. Although in colostrum samples we detected a greater number of anaerobic than aerobic bacterial genera, the latter were present with a greater relative abundance as the number of total reads was higher than that of anaerobic bacteria. Interestingly, breast milk contains high levels of oxygen, similar to those detected in venous plasma, that can justify the greater abundance of aerobic bacteria [26].

Considering bacterial interactions within the colostrum, we observed a different microbiota distribution in C-section relative to vaginal delivery colostrum. The mode of delivery, also seemed to have a strong impact on the relationships existing between microorganisms and for this reason different bacterial *hubs* were detected. Only five *hubs* were shared between C-section and vaginal delivery colostrum samples, such as *Achromobacter*, *Rhodanobacter*, *Ruminococcus*, *Serratia* and *Staphylococcus.* However, these were linked to different bacterial nodes in relation to the mode of delivery. In the vaginal delivery colostrum, for instance, *Achromobacter* showed 16 connections to microorganisms of both environmental and human origins, while in C-section colostrum *Achromobacter* had only 5 connections to bacteria commonly associated with the human body. However, the real meaning of these interactions is not clear and they are still the object of much study. In both C-section and vaginal delivery colostrum networks, the *Staphylococcus hub* was directly linked to *Propionibacterium*, while *Ruminococcus* interacted with *Faecalibacterium* and *Sutterella*, outlining a potential common role of these microorganisms in colostrum, independent of the mode of delivery. In particular, *Propionibacterium* is able to induce *Staphylococcus aureus* aggregation and production of biofilm which is one of the main mechanisms by which staphylococci colonize biotic and abiotic surfaces [27]. Staphylococci are often found on catheters and medical devices where they are able to produce a biofilm and colonize the environment. Similarly, during lactation, mammary glands are constituted by a complex network of “catheter-like” ducts representing an optimal environment for staphylococcal colonization which is probably enhanced by the positive interaction with *Propionibacterium* spp. [28]. Considering the *Ruminococcus hub*, instead, its interaction with *Sutterella* and *Faecalibacterium* has not been well clarified, even if increased abundance of *Ruminococcus* and *Sutterella* has been observed in the feces of children with autism spectrum disorder, suggesting that these two microorganisms have a pivotal role in behavioral disorders acting on the gut-brain axis [29]. Conversely, an opposite trend was highlighted for *Faecalibacterium* and *Ruminococcus,* whose abundance was reduced in subjects affected by Crohn’s disease (CD). Takahashi et al. (2016) underlined the involvement of intestinal dysbiosis in CD and in particular the reduction of butyrate-producing bacteria, such as *Ruminococcus torques* and *Faecalibacterium prausnitzii* that act as positive modulators of intestinal microbiota [30]. Probably, the interaction between *Ruminococcus*-*Sutterella*-*Faecalibacterium* is fundamental for the homeostasis of colostrum microbiota, limiting the potential pathogenicity of *Sutterella* spp., enhancing at the same time the beneficial activity of *Faecalibacterium*.

## Conclusions

The present study demonstrates that the mode of delivery plays a pivotal role in modulating the microbiota of the colostrum. Not only the abundance of different bacterial genera but also microorganismal interactions (microbiota network) were significantly different between C-section and vaginal delivery colostrum. Obviously, numerous factors can influence the colostrum microbiota composition; lifestyle, dietary habits, and the physical characteristics of the mother are all important features that can potentially impact on the composition of the colostrum and mature milk.

## Methods

### Study population

This study involved 29 mothers, 15 who underwent vaginal delivery and 14 who delivered by C-section, who were recruited from the postnatal wards (Policlinico GB Rossi, Verona, Italy).

Participants were selected and included in the study according to the following criteria: (i) compliance with the study protocol; (ii) healthy infants; (iii) collection of colostrum within 3 days after birth. Also the following exclusion criteria were considered: (i) mothers taking immunosuppressive agents; (ii) mothers following an antibiotic therapy during lactation; (iii) significant maternal or infant illness, or major birth defects.

The sample collection and investigation were conducted following ethical approval by the hospital committee, in accordance with Italian standards (Ethical Committee of the Azienda Ospedaliera of Verona, Italy, approval No. 1288). Informed consent was obtained from all subjects. Information about mother and newborn pairs are shown in Table 1.

**Table 1:** Characteristics of mother-newborn pairs based on the two mode of delivery. Data are expressed as mean (±SD)

		C-section delivery (15 pairs)	Vaginal delivery (14 pairs)
Maternal age (yrs)	Mean (±SD)	32,62 ± 5,11	29,5 ± 4,45
Parity	Mean (±SD)	1,67 ± 0,82	1,64 ± 0,5
Gestational age (wks)	Mean (±SD)	38,73 ± 2,49	39,5 ± 1,56
Sex		10 males	10 Males
		5 females	4 Females
Birth weight (g)	Mean (±SD)	3281,67 ± 685,56	3298,33 ± 600,72

### Collection and processing of colostrum samples

One sample of colostrum was collected from each mother within 3 days postpartum. Samples were collected in sterile plastic tubes after the mother’s hands and areola area were decontaminated using a preservative-free soap. Samples were initially stored at 4 °C prior to being frozen at −20 °C within two hours of expression. In the Verona laboratory, the samples were thawed and centrifuged at 1500 x *g* for 15 min at 4 °C to separate the fat and the aqueous phase. Finally, samples were shipped under controlled conditions to the Laboratory of Clinical Microbiology, Milan, Italy.

### Bacterial DNA extraction and 16S gene sequencing

Total DNA was extracted from colostrum samples using a Milk DNA Extraction Kit (Norgen, Thorold, Canada) following the manufacturer’s instructions.

Partial 16S rRNA gene sequences were amplified using the 16S Metagenomics Kit (Life Technologies, Italy) designed for the specific analysis of complex bacterial populations using the Ion Torrent sequencing technology. The two primer sets used for the amplification amplify the corresponding bacterial hypervariable regions of the 16S region: primer set V2–4-8 and primer set V3–6, 7–9. The PCR conditions used were 10 min at 95 °C, 30 cycles of 30 s at 95 °C, 30 s at 58 °C and 20 s at 72 °C, followed by 7 min at 72 °C. Amplification was carried out using a SimpliAmp thermal cycler (Life Technologies, Italy), while the integrity of the PCR amplicons was analyzed by means of gel electrophoresis. Finally, DNA sequencing was performed as previously described using the Personal Genome Machine (PGM) (Life Technologies, Italy) [1].

After sequencing, individual sequence reads were filtered to remove low quality and polyclonal sequences. Sequences matching the PGM 3′ adaptor were also automatically trimmed. 16 rRNA sequences were then analyzed combining a Basic Local Alignment Search Tool (BLAST) alignment to the curated Greengenes database, which contains more than 400,000 records, with a BLAST alignment to the premium curated MicroSEQ ID database, a high-quality library of full-length 16S rRNA sequences.

### The auto contractive map

The microbiota bacterial network of human colostrum was identified using AutoCM, a complex mathematical network able to establish the hierarchy of variables within a specific dataset. The microbiological application of AutoCM that has been clearly described by Drago et al. (2017) [1]. Briefly, the AutoCM system is a fourth-generation unsupervised artificial neural network (ANN) that is able to outperform numerous unsupervised algorithms [1]. The system can highlights the natural links among variables with a graph based on minimum spanning tree (MST) theory, discovering hidden trends and associations among variables, as this algorithm is able to create a semantic connectivity map in which non-linear associations are preserved and explicit connection schemes are described. The final result is a map where hubs can be defined as variables with the maximum amount of connections in the map.

### Characterization of anaerobe/aerobe and environmental bacteria

To characterize bacteria identified in the colostrum microbiota by sequencing, we used the scientific literature (https://www.ncbi.nlm.nih.gov) and different online free tools to discriminate between anaerobe and aerobe bacteria, as well as identify environmental microorganisms. The aforementioned tools were:

http://www.gbif.org

http://www.bacterio.net

https://www.embl.de

http://www.genome.jp/kegg

### Statistical analysis

The biodiversity index (Shannon, Simpson and Chao) and statistical analyses were carried out using R V.3.3.1, for Windows. Non-parametric Kruskal-Wallis and Mann-Whitney tests were used to find significant differences in α diversity and microbial taxa. Adjustment for multiple testing was evaluated with Dunn’s post-hoc test. *P*-values below 0.05 were considered statistically significant.
